# MMP-2 siRNA Inhibits Radiation-Enhanced Invasiveness in Glioma Cells

This article has been retracted.

**DOI:** 10.1371/journal.pone.0020614

**Published:** 2011-06-16

**Authors:** Aruna Venkata Badiga, Chandramu Chetty, Divya Kesanakurti, Deepthi Are, Meena Gujrati, Jeffrey D. Klopfenstein, Dzung H. Dinh, Jasti S. Rao

**Affiliations:** 1 Department of Cancer Biology and Pharmacology, University of Illinois College of Medicine, Peoria, Illinois, United States of America; 2 Department of Pathology, University of Illinois College of Medicine, Peoria, Illinois, United States of America; 3 Department of Neurosurgery, University of Illinois College of Medicine, Peoria, Illinois, United States of America; The University of Chicago, United States of America

## Abstract

**Background:**

Our previous work and that of others strongly suggests a relationship between the infiltrative phenotype of gliomas and the expression of MMP-2. Radiation therapy, which represents one of the mainstays of glioma treatment, is known to increase cell invasion by inducing MMP-2. Thus, inhibition of MMP-2 provides a potential means for improving the efficacy of radiotherapy for malignant glioma.

**Methodology/Principal Findings:**

We have tested the ability of a plasmid vector-mediated MMP-2 siRNA (p-MMP-2) to modulate ionizing radiation-induced invasive phenotype in the human glioma cell lines U251 and U87. Cells that were transfected with p-MMP-2 with and without radiation showed a marked reduction of MMP-2 compared to controls and pSV-transfected cells. A significant reduction of proliferation, migration, invasion and angiogenesis of cells transfected with p-MMP-2 and in combination with radiation was observed compared to controls. Western blot analysis revealed that radiation-enhanced levels of VEGF, VEGFR-2, pVEGFR-2, p-FAK, and p-p38 were inhibited with p-MMP-2-transfected cells. TUNEL staining showed that radiation did not induce apoptosis in U87 and U251 cells while a significant increase in TUNEL-positive cells was observed when irradiated cells were simultaneously transfected with p-MMP-2 as compared to controls. Intracranial tumor growth was predominantly inhibited in the animals treated with p-MMP-2 alone or in combination with radiation compared to controls.

**Conclusion/Significance:**

MMP-2 inhibition, mediated by p-MMP-2 and in combination with radiation, significantly reduced tumor cell migration, invasion, angiogenesis and tumor growth by modulating several important downstream signaling molecules and directing cells towards apoptosis. Taken together, our results demonstrate the efficacy of p-MMP-2 in inhibiting radiation-enhanced tumor invasion and progression and suggest that it may act as a potent adjuvant for radiotherapy in glioma patients.

## Introduction

Patients with glioblastoma multiforme (GBM), the most common type of human primary brain tumor and the most lethal of all human tumors, have a median survival of less than one year [1]–[3]. Despite advances in neurosurgery, radiation therapy, and chemotherapy, this prognosis has not changed significantly over the past two decades. Contributing to the deadly nature of the disease is the ability of glioblastoma cells to extensively invade normal brain tissue, thereby preventing a surgical cure and resistance of glioblastoma to existing therapeutic modalities, including radiotherapy [1]. Excessive proliferation, disseminated tumor growth, resistance to apoptotic stimuli, neovascularization, and suppression of anti-tumor immune surveillance are key biological features that contribute to the malignant phenotype of gliomas [4], [5]. Tumor cells obtain these invasive properties primarily because of their ability to secrete and activate proteolytic enzymes, such as serine, metallo, and cysteine proteases, which are capable of degrading extracellular matrix (ECM) components and breaking down other natural barriers to tumor invasion [6], [7].

Matrix metalloproteinases (MMPs) are zinc-dependent, proteolytic endopeptidases involved in cancer progression. Elevated levels of MMPs, in particular increased expression and activity of MMP-2 (72-kDa gelatinase A) and MMP-9 (92-kDa gelatinase B), have been correlated with an increased grade of glioma malignancy [8]–[10]. MMP-2 is highly expressed in gliomas as compared to normal brain tissue, and multiple roles have been indicated for this molecule in tumor progression. MMP-2 activates several key molecules leading to rapid cellular proliferation, increased motility, invasion, and angiogenesis of gliomas. Growth factor receptors, cell adhesion molecules, apoptotic ligands, angiogenic factors, chemokines, and cytokines are some of the diverse substrates targeted by MMPs [9], [11].

One of the major limitations in the treatment of glioma is the high prevalence of acquired resistance to radiation, which is likely associated with intrinsic cellular radioresistance, rapid cellular proliferation, and high invasiveness [12], [13]. Because radiation therapy continues to be the mainstay of cancer treatment, tumor resistance to ionizing radiation has been extensively studied. Of major interest is the role of MMPs in changing tumor cell properties and inducing an invasive phenotype after ionizing radiation [13]–[16]. Ionizing radiation induces an increase in MMP-2 levels in almost all human cancer types [17]–[23]. Radiation-enhanced expression as well as activation of the MMP-2 proteolytic system elevate or modify the bioavailability of several molecules that promote tumor progression. Enhanced MMP-2 secretion may increase tumor survival by decreasing apoptosis, stimulating proliferation, and increasing angiogenic and invasive potential. All these factors may contribute to the high vascularity as well as the high radioresistance of GBM [13]–[16].

There is strong biological background for the development of strategies targeting MMP-2. Nevertheless, several MMP inhibitors have proved to be disappointing in clinical trials due to either lack of benefits or major adverse effects [24]. Today, RNA interference-based, targeted silencing of gene expression is a strategy of potential interest for cancer therapy [25], [26]. Further, the specificity and potency of siRNA-MMP-2 in cell culture and in animal studies suggests that it has the potential to be a powerful therapeutic agent [27]–[29]. Viral vectors, particularly adenoviral ones, have been the primary gene transfer vehicle of choice. However, two concerns are the ability of adenoviral proteins to trigger an immune response and the limited length of time that the gene expression can be maintained in the target cells. Plasmid-based vectors have been considered to be more safe and efficient [30].

Since radiation is standard treatment for patients with GBM and because radiation-induced changes in invasive phenotype of glioma have been shown to be possibly due to changes in MMP activation, in the present study, we have tested the ability of a plasmid vector-mediated MMP-2 siRNA to modulate the ionizing radiation-induced invasive phenotype in human glioma cell lines, U-251 and U-87. We also investigated the anti-tumor effects of combining MMP-2 inhibition using the plasmid vector-mediated MMP-2 siRNA with radiation therapy *in vivo*. Our study shows that MMP-2 inhibition, mediated by plasmid DNA, in combination with radiotherapy reduces cell proliferation, tumor cell migration, invasiveness, and angiogenesis. We also show that inhibition of radiation-enhanced MMP-2 modulated important downstream signaling molecules, thereby directing the cells towards an apoptotic phenotype.

## Results

### p-MMP-2 transfection inhibits radiation-enhanced MMP-2 expression and cell viability

To examine the effect of radiation on MMP-2 expression, we determined MMP-2 activity in U-251 and U-87 cells irradiated with various X-ray doses. Radiation-induced MMP-2 activity increased up to 10 Gy for U-251 and up to 8 Gy for U-87 and decreased thereafter. The decreased levels of MMP-2 activity beyond 10 and 8 Gy for the two cell lines could be due to severe damage of DNA and other proteins. Maximal induction in pro-MMP-2 activity (72 kDa) was observed at 8 and 10 Gy when compared to the control, 0 Gy (Fig. 1A). Since MMPs play a role in the induction of malignant phenotype, we used a plasmid vector carrying siRNA against MMP-2 (p-MMP-2) to inhibit MMP-2 expression. We first determined the concentration of the plasmid DNA, which would give maximum inhibition of MMP-2 activity and levels when U-251 and U-87 cells were transfected. Figure 1B demonstrates that pro-MMP-2 activity was minimal when cells were transfected with 2 µg of the plasmid DNA. The figure shows a dose-dependent decrease in cellular MMP-2 levels with little or no MMP-2 detected when cells were transfected with 2 µg of the plasmid DNA. We therefore used this concentration (2 µg) of the plasmid DNA carrying MMP-2 siRNA or the scrambled sequence in combination with various doses of radiation for all experiments in the study. Western blots of cell lysates showed unchanged levels of MMP-9 when compared to the internal control GAPDH, thereby demonstrating the specificity of p-MMP-2. We next determined the effect of p-MMP-2 on radiation-induced MMP-2 expression. Figures 2A and B show pro-MMP-2 activity levels and protein levels, and mRNA levels of U-251 and U-87 transfected with p-MMP-2 or p-SV alone or in combination with various doses of radiation. Cells that were transfected with p-MMP-2 without radiation showed a significant decrease in activity/levels of MMP-2 when compared to the mock or p-SV controls or when compared to cells subjected to irradiation alone. The combination of p-MMP-2 and radiation caused a further decrease in MMP-2 levels. Maximal inhibition was observed with 6 Gy followed by 4 Gy. We further confirmed these results by immunofluorescence staining of the cells, which revealed similar results. There was a marked reduction in MMP-2 staining in all irradiated and concomitantly transfected cells, as well as in cells treated with p-MMP-2 alone (Fig. 2C). Cell viability/proliferation, as measured by MTT assay, was significantly reduced when U-251 and U-87 cells were concomitantly transfected with p-MMP-2 and irradiated or when cells were treated with p-MMP-2 alone when compared to the controls (Fig. 2D).

**Figure 1:** Radiation enhances MMP-2 and p-MMP-2 inhibits MMP-2 activity and expression in glioma cell lines. **A,** U-251 and U-87 cells were irradiated with 0–12 Gy X-ray, incubated for 24 h, and conditioned medium collected. MMP-2 activity was determined by gelatin zymography. The band intensities of MMP-2 activity were quantified by densitometry. *Columns*: mean of triplicate experiments; *bars*: SD; *p<0.01, **p<0.001, significant difference from non-irradiated (0 Gy) conditioned medium. **B,** U-251 and U-87 cells were transfected with mock (PBS), p-SV or p-MMP-2 (1, 2 or 3 µg). After 72 h of incubation, conditioned media was used to determine MMP-2 activity by gelatin zymography, and total cell lysates were used to determine MMP-2 and MMP-9 levels by Western blotting. The band intensities of MMP-2 activity as well as MMP-2 and MMP-9 protein levels were quantified by densitometry and normalized with the intensity of the mock bands. Glyceraldehyde-3-phosphate dehydrogenase (GAPDH) served as a loading control. *Columns*: mean of triplicate experiments; *bars*: SD; *p<0.01, **p<0.001, significant difference from mock or p-SV.

**Figure 2:** p-MMP-2 transfection inhibits radiation-enhanced MMP-2 activity and expression levels as well as cell viability. **A,** U-251 and U-87 cells were transfected with mock (PBS), p-SV or p-MMP-2 (2 µg), and after 72 h of incubation, cells were irradiated with 0, 2, 4, 6 or 8 Gy and incubated for a further 24 h. Conditioned media was used to determine MMP-2 activity by gelatin zymography, and total cell lysates were used to determine MMP-2 levels by Western blotting. **B,** Total RNA was used to determine MMP-2 mRNA transcription levels by RT-PCR with gene-specific primers. GAPDH served as a loading control. **C,** U-251 and U-87 cells were transfected with mock, p-SV or p-MMP-2 and irradiated as described above. 24 h after radiation, the cells were fixed and processed to visualize MMP-2 expression. The cells were mounted using mounting media with DAPI to visualize the nucleus. **D,** U-251 and U-87 cells were transfected with mock, p-SV or p-MMP-2, and irradiated for 72 h after transfection. After a another 24 h of incubation, cell viability was analyzed by MTT assay (absorbance read at 550 nm). *Columns*: mean of triplicate experiments; *bars*: SD; *p<0.01, significant difference from mock, p-SV or irradiated controls.

### p-MMP-2 inhibits radiation-enhanced glioma cell migration and invasion

Since MMP-2 has been implicated as an important factor in malignant glioma cell migration and invasion into the surrounding normal tissue, which is a major problem for any therapeutic modality, we studied the effect of p-MMP-2 on these processes. Since tumor spheroids mimic tumor growth, we allowed U-87 or U-251 cells to form spheroids, and then transfected and irradiated the cells. We observed a significant reduction in the migrating potency of cells transfected with p-MMP-2 and of cells that were concomitantly transfected and irradiated as compared to the controls. Cell migration was decreased five-fold and even more (particularly with 4 and 6 Gy) in the p-MMP-2 transfected and irradiated cells when compared to controls (Fig. 3). Matrigel invasion assay showed a significant inhibition of invasion by tumor cells that were transfected with p-MMP-2 without exposure to radiation and an even more significant dose-dependent inhibition when cells were concomitantly transfected and irradiated at various doses. Maximal inhibition was observed with 4 Gy followed by 6 Gy. Inhibition was significant when compared to mock or p-SV-transfected controls or to cells that were only subject to radiation. The normalization of the values as a percentage of the control (100%) cells treated with p-MMP-2 and concomitantly irradiated (6 Gy) showed a more than 90% inhibition (Fig. 4).

**Figure 3:** p-MMP-2 transfection in combination with radiation inhibits glioma cell migration. U-251 and U-87 cells were cultured for formation of spheroids as described in Materials and Methods. Spheroids were then transfected with mock, p-SV or p-MMP-2, and followed by irradiation as described earlier. At the end of the migration assay, spheroids were fixed and stained with Hema-3. Migration of cells from spheroids to monolayers was measured using a microscope calibrated with a stage and ocular micrometer. *Columns*: mean of triplicate experiments; *bars*: SD; *p<0.01, **p<0.001, significant difference from mock, p-SV or irradiated controls.

**Figure 4:** p-MMP-2 transfection inhibits radiation-enhanced glioma cell invasion. U-251 and U-87 cells were transfected with mock, p-SV or p-MMP-2, and irradiated as described earlier. Cells were trypsinized and counted, and 5×10^5^ cells from each treatment condition were allowed to invade transwell inserts containing 12-µm-pore polycarbonate membranes pre-coated with Matrigel for 24 h at 37°C. Afterwards, cells were fixed and stained with Hema-3. Cells that had migrated to the lower side of the membrane were photographed under a light microscope at 20× magnification. Percentages of invading cells were quantified by counting five fields from each treatment condition. *Columns*: mean of triplicate experiments; *bars*: SD; *p<0.01, **p<0.001, significant difference from mock or irradiated controls.

### p-MMP-2 inhibits tumor-induced and radiation-enhanced angiogenesis *in vitro* and decreases expression of angiogenesis-associated molecules

We next determined the ability of p-MMP-2 to inhibit angiogenesis. Glioblastoma is one of the most highly angiogenic tumors; MMP-2 is an important angiogenic molecule that promotes tumor vascularization, in turn rendering the tumor cells resistant to radiotherapy. Conditioned media from p-MMP-2-treated alone or in combination with radiation treated U-87 or U-251 cells failed to induce capillary-like formation when added to cultured human microvascular endothelial cells (HMECs) in contrast to conditioned media obtained from control and p-SV transfected cells, which was capable of triggering the angiogenic process. Mock and p-SV treated cells that were subject to radiation demonstrated enhanced angiogenesis, as is evident from the increase in percentage of branching when compared to their non-irradiated counterparts (Fig. 5A). Western blot analyses revealed enhanced levels of vascular endothelial growth factor (VEGF), a well-known inducer of angiogenesis, VEGF receptor-2 (VEGFR-2), and also a corresponding increase in phosphorylation of VEGFR-2 in lysates of irradiated glioma cells. p-MMP-2 treatment markedly reduced radiation-enhanced protein levels, which were almost completely inhibited when cells were simultaneously treated with the MMP-2 inhibitor and irradiated at 4 or 6 Gy (Fig. 5B). We also demonstrated the effect of radiation and the combined treatment on p38 and FAK, which are downstream molecules of VEGF signaling. Radiation-enhanced levels of phosphorylated p38 and phosphorylated FAK were largely inhibited when cells were simultaneously transfected with p-MMP-2. Levels of total p38 and FAK remained unchanged for the different treatment groups, when compared to the internal GAPDH control (Fig. 5B).

**Figure 5:** p-MMP-2 inhibits radiation-enhanced tumor culture medium-induced microtubule network formation in endothelial cells and downregulates expression of angiogenesis-associated molecules. **A,** Human microvascular endothelial cells (5×10^4^) were seeded in 96-well plates and cultured with conditioned medium collected from U-251 and U-87 glioma cells transfected with mock, p-SV, and p-MMP-2, and irradiated as described earlier. 24 h after radiation treatment, the cells were washed, fixed and stained with Hema-3 and photographed. Percentages of branches were quantified by counting five fields in each condition. *Columns*: mean of triplicate experiments; *bars*: SD; *p<0.01, **p<0.001, significant difference from mock or irradiated controls. **B,** U-251 and U-87 transfection and radiation was carried out as described earlier. 24 h after radiation, whole cell lysates were prepared and analyzed by Western blotting for the angiogenic molecules VEGF, VEGFR-2 and p-VEGFR-2 as well as p-FAK, FAK, p-p38 and p38. GAPDH served as a loading control.

### p-MMP-2 inhibits colony formation and induces apoptotic cell death in irradiated glioma cells

We performed the colony forming assay to determine the effect of p-MMP-2 and radiation on the survival of glioma cells. Treatment with p-MMP-2 followed by irradiation as well as treatment with p-MMP-2 alone significantly reduced clonogenic survival when compared to the irradiated cells (Fig. 6A). High levels of MMP-2 in gliomas and radiation-enhanced MMP-2 are known to render tumor cells less susceptible to apoptosis. TUNEL staining showed that radiation did not induce apoptosis in the glioma cells while a significant increase in TUNEL-positive cells was observed when irradiated cells were simultaneously transfected with p-MMP-2 as compared to the controls. Quantification revealed up to 80% induction of apoptosis in cells treated with the MMP-2 siRNA construct and irradiated at 6 Gy (Fig. 6B). Moreover, caspases 3, 8 and 9, which mediate the apoptotic mechanism, were cleaved and activated in irradiated cells transfected with p-MMP-2 as shown by comparison of Western blot analysis of cell lysates from the different treatment groups (Fig. 6C).

**Figure 6:** p-MMP-2 inhibits colony formation and induces apoptosis and activation of pro-apoptotic molecules in glioma cells. **A,** Clonogenic assay was performed as described in Materials and Methods. The cells were cultured, and colonies larger than 50 cells were counted. *Columns*: mean of triplicate experiments; *bars*: SD; *p<0.01, significant difference from radiation. **B,** U-251 and U-87 cells were transfected with mock, p-SV or p-MMP-2, and irradiated as described earlier. After 24 h of radiation, cells were evaluated with the TUNEL assay according to manufacturer's instructions and photographed under fluorescent microscopy. Apoptosis was measured by counting the percentage of cells that showed DNA staining in five different fields in each group. *Columns*: mean of triplicate experiments; *bars*: SD; *p<0.01, **p<0.001, significant difference from mock, p-SV or irradiated controls. **C,** Equal amounts of protein from whole cell lysates of control and treated cells were analyzed by Western blotting using caspase-specific primary antibodies. GAPDH served as a loading control.

### p-MMP-2 combined with radiation inhibits tumor growth *in vivo*

For the intracerebral injections, we chose the glioblastoma cell line U-251, which forms highly invasive tumors in athymic mice in contrast with U-87 cells that form solid and well defined tumors. Ten days after tumors were induced, animals were treated on alternate days for a total of 4 doses with 60 µg per dose of p-SV or pMMP-2 or phosphate-buffered saline (mock). Mice were injected with stably transfected U-251 cells expressing a luciferase plasmid, which enabled us to monitor tumor growth by intraperitoneally injecting D-luciferin into the animals. Over a 6-week period, tumor growth was predominantly inhibited in the animals treated with p-MMP-2 alone or in combination with radiation when compared with the mock or p-SV controls as observed in the IVIS images and subsequently confirmed by hematoxylin and eosin (H&E) staining of the tumor sections (Figs. 7A–B). Control animals developed symptoms of weight loss and neurological degradation before they were euthanized, whereas animals treated with p-MMP-2 alone or concomitantly irradiated remained symptom-free. No significant differences were observed between animals treated with mock or p-SV in terms of tumor size or symptoms. Brain sections were analyzed for expression of MMP-2 by immunohistochemistry (Fig. 8A). Mice treated with p-MMP-2 alone or in combination with radiotherapy showed a decrease in MMP-2 expression. Conversely, in control and p-SV treated mice or even mice that were subject to only radiation in which MMP-2 expression was detected mostly at the invasive edge of the tumor and in cells surrounding the necrotic areas as well as reactive endothelial cells within and around the tumor area. Confirming the *in vitro* findings, VEGF and pFAK were also suppressed in the animals treated with MMP-2 siRNA alone or in combination with radiation (Fig. 8A). TUNEL staining of tissue sections showed that radiation did not induce apoptosis in the glioma cells while predominant TUNEL staining was observed in tissues of mice that were treated with p-MMP-2 alone and in those that were concomitantly irradiated (Fig. 8B). Further, we noticed that the invasiveness of the tumor cells into adjacent normal brain tissue of mice increased with radiation compared to mock and pSV controls, but decreased in mice that received p-MMP-2 alone or in combination of radiation (Fig. 8C). Further, tumor infiltrating cells were detected in non-tumor regions of brain sections from mice using Human nuclei (HuNu) antibody, a histological marker for identification of human cells (a specific human nuclear antigen). A considerable number of tumor infiltrating cells were observed in tumor sections from mice that received mock and pSV treatments. In addition, we observed a significant increase in the number of tumor infiltrating cells in tumor sections from mice that received radiation treatment. However, we observed a drastic reduction in radiation-induced tumor cell infiltration in tumor sections from mice that received pMMP-2 (Fig. 8D). The immunoreactivity of MMP-2 in tumor sections from mice that received both radiation and p-MMP-2 treatments also showed that p-MMP-2 inhibited radiation-induced MMP-2 expression. These results suggest that p-MMP-2 could serve as an adjuvant with low-dose radiation therapy against glioblastoma.

**Figure 7:** p-MMP-2 combined with radiation inhibits tumor growth *in vivo*. U-251 (1×10^6^) cells were injected intracerebrally into athymic mice. After ten days, animals were separated into five groups and were treated on alternate days with intracerebral injections of p-SV or p-MMP-2 for a total of 4 doses (60 µg per dose) and 2 doses of radiation (4 Gy per dose) as described in Materials and Methods. Six weeks after the experiment was initiated, mice were euthanized with intracardiac perfusion of PBS, followed by formaldehyde. The brains were then removed. **A,** Six weeks after the experiment was initiated, an intraperitonal injection of 2.5 mg D-luciferin sodium salt diluted in 50 µL of PBS was given, and animals were photographed under the IVIS camera for fluorescent light emission. The brains were removed and fixed in 10% phosphate-buffered formaldehyde, and the fixed tissue samples were then processed into paraffin blocks. Brain sections (5 µM thick) were stained with hematoxylin and eosin (H&E), and photographed under a light microscope (4× and 40×). **B,** Every fifth or sixth brain section (5 µM thick) was stained with H&E solution, and the tumor masses (H&E-stained) were manually traced on the microscope attached computer screen. Areas were calculated using Image Pro Discovery Program software (Media Cybernetics, Inc., Silver Spring, MD). The total tumor volume was calculated as the summed area on all slices, multiplied by the slice separation. *Columns*: mean of area of tumor portion of all mice in the group (n = 8); *bars*: SD; *p<0.01, **p<0.001, significant difference from mock, p-SV or irradiated controls.

**Figure 8:** p-MMP-2 combined with radiation enhances apoptosis *in vivo*. **A,** Immunohistochemical analysis of brain sections using anti-MMP-2, anti-VEGF and anti-pFAK antibodies. Sections were photographed (60×). Also shown is the negative control where the primary antibody was replaced by non-specific IgG (insets). **B,** Tissue sections of mice were evaluated with the TUNEL assay according to manufacturer's instructions and photographed under fluorescent microscopy (60×). For the negative control, samples were incubated with label solution (without terminal transferase) instead of TUNEL reaction mixture (insets). **C,** siRNA against MMP-2 inhibits U251 tumor cell invasion *in vivo*. H&E staining was performed according to standard protocol, and representative pictures of tumor sections from mock, pSV, p-MMP-2-treated mice are shown (20× and 60×). **D**, Immunohistochemical analysis of brain sections using anti-human nuclei (HuNu) antibody, a histological marker for identification of human cells (a specific human nuclear antigen). Entire brain sections were photographed (4×; middle row); shown on the top row is a non-tumor region (40×; top row); and shown on the bottom row is tumor and non-tumor overlapping region (40×; bottom row). Also shown is the negative control where the primary antibody was replaced by non-specific IgG (inset).

## Discussion

Findings of the present study demonstrate the anti-tumor efficacy of combining a plasmid vector-mediated MMP-2 inhibitor (p-MMP-2) with ionizing radiation to target radiation-induced invasiveness and angiogenesis in glioma cells. Our results show that p-MMP-2 significantly inhibited radiation-enhanced MMP-2 protein expression and activity and its associated tumorigenic properties, such as cell proliferation, tumor cell migration, invasion, and angiogenesis in two human glioma cell lines, U-251 and U-87. We also show that the decrease in MMP-2 expression/activity further modulated important downstream signaling molecules directing the cells towards an apoptotic phenotype when administered in combination with radiotherapy.

MMP-2 activation has been associated with invasive phenotype in glioma cells [31]–[33]. In our experiments, the MMP-2 inhibitor, p-MMP-2, significantly downregulated MMP-2 protein expression and activity and modulated multiple biological behaviors that determine the malignant progression of gliomas. Previous reports show that ionizing radiation increased MMP-2 activity and protein secretion along with invasiveness of glioma cells [15]. We observed that ionizing radiation induced a dose-dependent increase in MMP-2 activity in U-251 and U-87 cells. As demonstrated by Wick, et al., [34] we also observed that irradiation promoted the accumulation of MT1-MMP and loss of TIMP-2 protein, possibly shifting the balance of these molecules in favor of MMP-2. Treatment of cells with p-MMP-2 and in combination with irradiation seemed to show a slight, though not significant, decrease in levels of MT1-MMP and more or less unchanged levels of TIMP-2 when compared to irradiated cellular protein levels (data not shown). This was of interest as the activation and regulation of MMP-2 is closely associated with MT1-MMP and TIMP-2. Given the specificity of our p-MMP-2 siRNA and its ability to significantly downregulate radiation-enhanced invasiveness, angiogenesis, and cell survival, it is very evident that MMP-2 might be associated with the exceeding invasiveness after radiation. Several studies have shown that MMP-2 and MMP-9 promote cancer progression by increasing tumor cell growth, migration, invasion, metastasis, and angiogenesis [7], [31], [32], [35], [36]. Thus, following radiation, it is logical that the elevated levels of MMP-2 and a subsequent increase in activation of the MMP-2 proteolytic system would only lead to enhanced invasiveness. MMPs exert these effects by cleaving a diverse group of substrates, which include not only structural components of the extracellular matrix, but also growth factor binding proteins, growth factor precursors, receptor tyrosine kinases, cell adhesion molecules, and other proteinases [9]. There was a marked increase in VEGF and VEGFR-2 secretion and an increase in phosphorylated VEGFR-2 after irradiation of glioma cells, which was almost completely inhibited by p-MMP-2 treatment. Radiation therapy plays a role in upregulating the expression of molecules such as VEGF, VEGFR, and EGFR [37]–[39], all of which are considered key targets for novel anti-cancer therapies [40], [41]. Further, studies support a possible link between MMP-2 and the potent angiogenic factor, VEGF. MMPs may stimulate VEGF release from tumor cells either directly or by activating factors involved in VEGF release or by mobilizing VEGF from the extracellular compartments [42]–[44]. Thus, by decreasing the availability of VEGF, MMP-2 downregulation efficiently blocked radiation-enhanced angiogenesis in U-251 and U-87 cells in the present study. Several studies demonstrated a marked increase in VEGF secretion following irradiation of cancer cells [15]. Kaliski, et al. [45] showed that irradiated melanoma cells displayed enhanced invasive capacity with increased MMP-2 expression and subsequently induced VEGF protein secretion. Specific MMP-2 inhibition blocked VEGF upregulation and inhibited tumor growth and angiogenesis *in vivo*. Hovinga, et al. [46] showed that radiation-enhanced VEGF secretion increased angiogenesis and decreased apoptosis, both leading to GBM radioresistance. As a consequence of VEGF signaling, many proteins are activated by VEGFR-2 via an unknown mechanism; these proteins include Src, phosphoionisitide 3-kinase (PI3K), focal adhesion kinase (FAK), and p38 mitogen activated protein kinase (p38 MAPK). These downstream signal transduction molecules propagate a signal leading to several different endothelial cellular functions such as survival, permeability, migration, and proliferation [47]. In the present study, concomitant with the decrease in VEGF and VEGFR-2, p38 and FAK phosphorylation were also downregulated, with a corresponding inhibition of tumor cell migration and invasiveness. Radiation-enhanced VEGF has also been shown to induce anti-apoptotic pathways and thereby promote tumor growth after irradiation. VEGF is reported to reduce apoptosis after irradiation in human leukemia cells and in human and murine mammary adenocarcinoma cells [48]–[50]. The simultaneous administration of p-MMP-2 with radiation opposed the anti-apoptotic phenotype and led to cleavage/activation of the pro-apoptotic molecules caspase 3, caspase 8 and caspase 9. Studies have shown that virtually all glioma-derived cell lines exhibit resistance to radiation and do not undergo radiation-induced primary apoptosis [51], [52]. In the present study, U-251 and U-87 cells demonstrated very high levels of apoptosis as shown by TUNEL assay when irradiated cells were concomitantly administered p-MMP-2. These findings were further validated *in vivo*. In our *in vivo* studies, p-MMP-2 reduced tumor size by more than 80% compared to mock or pSV. Although the tumor size in mice that received radiation treatment alone did not increase significantly, the invasive nature of the tumor did increase drastically. Tumor cells that manage to escape the lethal effects of irradiation often adapt more aggressive properties, proliferate more rapidly and display enhanced migratory, invasive and angiogenic potential [53], [54]. Further, sub-lethal doses of radiation have a toxic effect on healthy tissues and may also result in a more aggressive and malignant tumor due to the development of resistant cancer cell sub-populations that have enhanced proliferative, invasive and angiogenic properties [54]. Treatment with both p-MMP-2 and radiation did reduce radiation-induced tumor cell infiltration and tumor size by ∼80% compared to mock and pSV controls (Figs. 7A–B).

Radiation-enhanced expression as well as activation of the MMP-2 proteolytic system elevate or modify the bioavailability of several molecules that promote tumor progression [17]–[23]. Further, enhanced MMP-2 may increase tumor survival by decreasing apoptosis, stimulating proliferation, and increasing angiogenic and invasive potential [13]–[16]. Since the downregulation of MMP-2 seems to cause the modulation of several other molecules and pathways, MMP-2 siRNA is effective in modulating radiation-enhanced molecules, invasiveness and altering signaling pathways, thereby driving the cells through apoptosis.

It is worth noting that in all of our experiments, glioma cells that were treated only with p-MMP-2 showed a significant downregulation of tumorigenic properties and were capable of acquiring an apoptotic phenotype. This proves the anti-tumor efficacy of p-MMP-2. Nevertheless, since radiotherapy is the standard treatment for glioma and malignant glioma is one of the most radioresistant tumor types, the administration of p-MMP-2 prior to radiotherapy could be a potent adjuvant therapeutic approach to improve the efficacy of radiotherapy for glioma. Adenoviral vectors have been widely used both in cells and *in vivo* for the delivery of MMP-2 siRNA [27]–[29]. Although they may be capable of efficiently delivering the gene to the target cells, adenovirus carries the risk of triggering an immune response, which limits the length of time that the gene expression can be maintained in the target cells. Plasmids, on the other hand, being non-infectious and non-immunogenic, could be much safer and provide stability of gene transfer [30]. The results of our study demonstrated the efficacy of p-MMP-2 in inhibiting radiation-enhanced tumor invasion and progression and suggest that it may act as a potent adjuvant for radiotherapy in malignant glioma.

## Materials and Methods

### Ethics Statement

The Institutional Animal Care and Use Committee (IACUC) of the University of Illinois College of Medicine at Peoria, Peoria, IL, USA, approved all surgical interventions and post-operative animal care. The consent was written and approved. The animal protocol number is 858, dated May 27, 2009, and renewed on April 27, 2010.

### Cell cultures

Glioblastoma cell lines U-251 and U-87 obtained from American Type Culture Collection (ATCC, Manassas, VA) were grown in Dulbecco's modified Eagle's medium (DMEM). Cultures were supplemented with 1% glutamine, 100 µg/mL streptomycin, 100 U/mL penicillin and 10% fetal calf serum (FCS) and maintained in a humidified atmosphere containing 5% CO_2_ at 37°C.

### Plasmid vector constructs, transient transfection, and radiation treatment

The plasmid constructs carrying siRNA against MMP-2 (p-MMP-2) and a scrambled MMP-2 sequence (p-SV) were designed and constructed as previously described [27]. pcDNA3.0 (Invitrogen) with a CMV promoter was used for the construction of vectors. The following siRNA sequences were cloned into the pcDNA3.0: aacggacaaagagttggcagtatcgatactgccaactctttgtccgtt for p-MMP-2 inverted repeat sequence and gcacggaggttgcaaagaataatcgattattctttgcaacctccgtgc for p-SV inverted repeat sequence. Annealed oligos were sequentially ligated to pcDNA3.0 at the *Nhe* I site. Briefly, 150,000 cells were seeded in 6-cm diameter dishes and grown in DMEM supplemented with 10% FCS. The cells were transfected with mock (PBS), p-SV, or p-MMP-2. Transfections were performed using FuGENE *HD* transfection reagent (Roche Applied Science, Indianapolis, IN) as per the manufacturer's instructions. After 72 h of transfection, cells were irradiated with a single dose of radiation (2, 4, 6, 8, 10 or 12 Gy). The RS 2000 Biological irradiator (Rad Source Technologies, Boca Raton, FL) X-ray unit operated at 150 kv/50 mA was used for radiation treatments. All experiments were performed 24 h after radiation.

### Gelatin zymography

Cells were transfected with mock, p-SV or p-MMP-2 alone or in combination with various single doses of radiation (2, 4, 6, 8, 10 or 12 Gy) to which cells were exposed 72 h after transfection. Following radiation, cells were cultured for 24 h in serum-free DMEM/F-12 medium. The serum-free conditioned medium was collected and equal amounts of protein were used to determine MMP-2 activity. Gelatin zymography was performed as previously described [55].

### Reverse transcription-PCR

Cells were transfected and irradiated as described above. Total RNA was extracted using TRIZOL reagent (Life Technologies, Rock-ville, MD) according to the manufacturer's protocol. RT-PCR was performed as described previously [27]. PCR products were resolved on 2% agarose gels and were visualized by ethidium bromide staining. To normalize for the amount of input RNA, RT-PCR was performed with primers for *GAPDH*. We used the following specific primers: *MMP-2*, forward 5′-GTGCTGAAGGACACACTAAAGAAGA-3′, and reverse 5′-TTGCCATCCTTCTCAAAGTTGTAGG-3′; *GAPDH*, forward 5′-TGAAGGTCGGAGTCAACGGATTTGGT-3′, and reverse 5′-CATGTGGGCCATGAGGTCCACCAC-3′. Images were generated by Alpha Innotech Image Acquisition and Analysis Software.

### Western blot analysis

U-251 and U-87 cells were transfected and irradiated as described earlier. Equal amounts of total protein from cell lysates obtained by lysing cells in a suitable buffer [50 mM/L Tris-HCl (pH 7.4), 150 mM/L NaCl, 1% IGEPAL, 1 mM/L EDTA, 0.25% sodium deoxycholate, 1 mM/L sodium fluoride, 1 mM/L sodium orthovanadate, 0.5 mM/L PMSF, 10 µg/mL aprotinin, 10 µg/mL leupeptin] were separated by SDS–PAGE and transferred to polyvinylidene difluoride membranes (Bio-Rad, Hercules, CA). After blocking with 5% nonfat dry milk and 0.1% Tween-20 in PBS, membranes were incubated with 1∶1000 dilution of primary antibodies followed by incubation in HRP-conjugated secondary antibodies. Membranes were developed using the ECL system (Amersham Bioscience Corp., Piscataway, NJ). Primary antibodies used in this study were: MMP-2, MMP-9, VEGF, VEGFR-2, pVEGFR-2, pFAK, FAK, p-p38, total p38, caspase 3, caspase 8, caspase 9, GAPDH (used as a loading control), HRP conjugated secondary antibodies (Santa Cruz Biotechnology, SantaCruz, CA).

### Cell proliferation assay

Cell growth was assessed by MTT assay. U-251 and U-87 cells (5×10^3^ cells per well) were grown in 96-well plates, transfected and irradiated as described earlier. Proliferation rate was measured 24 h after treatment by adding 20 µL of MTT (3-(4,5-dimethylthiazol-2-yl)-2,5-diphenyltetrazolium bromide) solution (R&D Systems, Minneapolis, MN) to each well and further incubating the plate for 1 h. Samples were read on a microplate reader using test wavelength of 550 nm and reference wavelength of 655 nm.

### Immunofluorescence

U-251 and U-87 cells were cultured in 8-well chamber slides (Nalge Nunc International, Naperville, IL) (10^4^ cells per well), transfected and irradiated as described earlier. After 24 h of treatment, cells were fixed in 3% formaldehyde and incubated with 0.2% Triton X-100 in PBS. Cells were then blocked with 3% bovine serum albumin (BSA) for 1 h and incubated with mouse anti-MMP-2 in 1% BSA in PBS (dilution 1∶500). Cells were washed with PBS and mouse fluorescein isothiocyanate (FITC)-conjugated secondary antibody was added for 1 h. Finally, slides were washed with PBS, mounted and examined under a fluorescent microscope connected to an Olympus camera.

### Spheroid migration assay

Cells (4×10^4^) were seeded in 96-well plates coated with 1% agarose in PBS and cultured on a shaker at 100 rpm for 48 h. After single spheroids formed, cells were transfected with mock, p-SV or p-MMP-2 alone or in combination with various doses of radiation as described earlier. Treated spheroids were placed in the center of each well of vitronectin-coated 96-well plates and were cultured at 37°C for 24 h in serum-free DMEM, after which they were fixed and stained with Hema-3. The migration of cells from the center of the spheroids to monolayers was measured using a microscope calibrated with a stage and ocular micrometer. We used Image Pro Discovery Program software to determine the index of cell migration (Media Cybernetics, Inc., Silver Spring, MD) as described previously [36].

### Matrigel invasion assay

U-251 and U-87 cells were transfected and irradiated as described earlier. Transwell inserts (ThinCertTM; Greiner Bio-One, Monroe, NC) with 8 µm pores were coated with 200 µL growth factor reduced Matrigel (Collaborative Research, Inc., Boston MA) at a concentration of 0.7 mg/mL in DMEM serum-free medium for 3–4 h. 500 µL of cell suspension (5×10^5^ cells) were added into wells in triplicate. Cells were allowed to invade through the Matrigel for 24 h. Cells in the upper chamber were removed by cotton swab. Cells adhered on the outer surface that had invaded though the Matrigel were fixed, stained with Hema-3, photographed and counted under a light microscope as previously described [36].

### *In vitro* angiogenesis assay

Conditioned medium-induced microtubule network formation *in vitro* was determined. Cells were transfected and irradiated as described earlier. Conditioned medium from U-251 and U-87 control and treated cells was collected and added to HMEC (5×10^4^ per well) seeded the previous day in 96-well plates. HMEC were incubated for 24 h and the formation of microtubule networks was examined after fixing and staining the cells with Hema-3. The angiogenic result was measured by counting the relative branch points in each field for the different treatment groups.

### Clonogenic assay

U-251 and U-87 cells were transfected and irradiated as described earlier. Cells were trypsinized and 200 cells were seeded in 100-mm Petri dishes. On day 10 after irradiation, cells were fixed in methanol and stained with Giemsa. Colonies (>50 cells) were counted and survival fraction was calculated as number of colonies divided by the number of plated cells.

### TUNEL assay and apoptosis

U-251 and U-87 cells were grown in 8-well chamber slides, transfected and irradiated as described earlier. Then, terminal deoxynucleotidyl transferase biotin-dUTP nick end-labeling (TUNEL) assay was performed using an apoptosis detection kit (Roche Applied Science, Indianapolis, IN) according to the manufacturer's instructions. Briefly, cells were fixed with 3% paraformaldehyde and incubated with 0.2% Tween-20, 0.2% BSA in PBS for 15 min at room temperature. Cells were washed with PBS and incubated with terminal deoxynucleotidyl transferase end-labeling cocktail for 60 min. The reaction was stopped with Tris-borate buffer, and cells were washed and incubated for 30 min in the dark with avidin-FITC solution diluted in the provided blocking buffer. Finally, cells were washed, mounted and photographed under a fluorescent microscope. Apoptosis was measured as the average percentage of positive nuclei per field for each treatment.

### Animal studies

Experiments in nude mice were carried out according to the protocol approved by the IACUC of this institution. U-251 glioblastoma cells stably transfected with a luciferin-expressing plasmid were grown in serum-containing culture media. Cells were trypsinized and resuspended in PBS. 10 µL (1×10^6^ cells) was injected intracerebrally into nude mice. To detect tumor growth, animals received an intraperitoneal injection of 2.5 mg of D-luciferin sodium salt (Gold Biotechnology, St Louis, MO) suspended in 50 µL of PBS, and tumor growth was monitored using IVIS-200 Xenogen imaging system (Xenogen Corporation, Alameda, CA). Tumors were allowed to grow for 10 days before animals were separated into five treatment groups of eight mice each. Two groups of animals were treated on alternate days with intracerebral injections of p-SV or p-MMP-2 for a total of 4 doses (60 µg per dose in 10 µL volume; flow rate ∼1 µL/10 sec). Between the first and the second injections and between the second and the third injections, the animals that were administered p-MMP-2 were also irradiated with a dose of 4 Gy each time. Another group of animals was subjected to only irradiation at 8 Gy. Only the tumor region was exposed to radiation while the rest of the mouse body was covered with lead sheet. Control animals were injected with PBS (mock) only. After 6 weeks and/or when the control animals started showing symptoms, animals were anesthetized and euthanized by intracardiac perfusion of PBS followed by formaldehyde. The brains were removed, and fixed in 10% phosphate-buffered formaldehyde and the fixed tissue samples were then processed into paraffin blocks. Every fifth or sixth section (5 µm thick) was stained with hematoxylin-eosin solution (H&E) and the tumor masses (H&E-stained) were manually traced on the microscope attached to a computer. Areas were calculated using Image Pro Discovery Program software (Media Cybernetics, Inc., Silver Spring, MD). The total tumor volume was calculated as the summed area on all slices, multiplied by the slice separation [56], and normalized to the volume of tumor in p-SV treated mice. For the immunohistochemical experiments, brain sections were deparaffinized in xylene and rehydrated through graded alcohol. Then, slides were incubated with 0.1% Triton X-100, blocked with 3% BSA in PBS, and incubated with anti-MMP-2, anti-VEGF, anti-pFAK (Santa Cruz Biotechnology, SantaCruz, CA) or anti-human nuclei (HuNu) antibody (Millipore, Temecula, CA) (1∶10 dilution). After a rinse in PBS, slides were incubated with HRP-conjugated secondary antibody for 1 h at a dilution of 1∶300, washed again with PBS and incubated with 0.05% 3,30-diaminobenzidine as chromogen. Finally, slides were counterstained with hematoxylin, mounted and observed under a light microscope. Tissue sections were also subject to TUNEL assay performed using an apoptosis detection kit (Roche Applied Science, Indianapolis, IN) according to the manufacturer's instructions.

### Statistical analysis

Data are presented as the arithmetic mean ± standard deviation (SD) of at least three independent experiments, each performed at least in triplicate. Results were analyzed using a two-tailed Student's t-test to assess statistical significance. In the animal experiments, the mean differences in tumor volumes were compared among treatment groups using a one-way analysis of variance (ANOVA). Statistical differences are presented at probability levels of p<0.05, <0.01 and <0.001.
